The article "Diagnosis of Alzheimer Disease Using 2D MRI Slices by Convolutional Neural Network" was retracted in 2023. Reasons: signs of a paper mill; suspected computer-generated content; unreliable results or conclusions; lack of ethics approval or compliance.

# Diagnosis of Alzheimer Disease Using 2D MRI Slices by Convolutional Neural Network

**DOI:** 10.1155/2021/6690539

**Published:** 2021-02-02

**Authors:** Fanar E. K. Al-Khuzaie, Oguz Bayat, Adil D. Duru

**Affiliations:** ^1^Graduate School of Science and Engineering, Altinbas University, Istanbul, Turkey; ^2^Department of Physical Education and Sports Teaching, University of Marmara, Istanbul, Turkey

## Abstract

There are many kinds of brain abnormalities that cause changes in different parts of the brain. Alzheimer's disease is a chronic condition that degenerates the cells of the brain leading to memory asthenia. Cognitive mental troubles such as forgetfulness and confusion are one of the most important features of Alzheimer's patients. In the literature, several image processing techniques, as well as machine learning strategies, were introduced for the diagnosis of the disease. This study is aimed at recognizing the presence of Alzheimer's disease based on the magnetic resonance imaging of the brain. We adopted a deep learning methodology for the discrimination between Alzheimer's patients and healthy patients from 2D anatomical slices collected using magnetic resonance imaging. Most of the previous researches were based on the implementation of a 3D convolutional neural network, whereas we incorporated the usage of 2D slices as input to the convolutional neural network. The data set of this research was obtained from the OASIS website. We trained the convolutional neural network structure using the 2D slices to exhibit the deep network weightings that we named as the Alzheimer Network (AlzNet). The accuracy of our enhanced network was 99.30%. This work investigated the effects of many parameters on AlzNet, such as the number of layers, number of filters, and dropout rate. The results were interesting after using many performance metrics for evaluating the proposed AlzNet.

## 1. Introduction

The normal brain of humans consists of mainly three regions, namely, white matter (WM), gray matter (GM), and cerebrospinal fluid (CSF) [1]. The white matter is called as such because of its white appearance. It contributes about sixty percent to the total brain volume. The gray matter is responsible of the whole processing of the neural signals. It consists of dendrites and the neuron nuclei. It contributes almost about forty percent of the total brain volume. Cerebrospinal fluid is a colorless fluid that provides protection from mechanical shocks and also emits some important hormones to make the communication possible among the white matter, gray matter, and spinal cord of the central nervous system [2]. It is known that the family of artificial intelligence (AI) includes many algorithms and methods which could be used in different aspects of our life, for example, genetic algorithm [3–5] and neural networks [6]. Machine learning (ML) is a field of artificial intelligence that usually employs factual procedures to allow PCs to “learn” by utilizing information from saved data sets. At a very basic level, deep learning (DL) is a machine learning subset [7]. Deep learning can be defined as a neural network which uses a huge number of parameters and layers. There are many fundamental network architectures [8] like (i) convolutional neural networks (CNNs) which are basically a standard neural network that has been extended across space using shared weights [9]. A convolutional neural network (CNN) is designed to recognize images by having convolutions inside, which see the edges of a recognized object on the image [10]. (ii) Recurrent neural networks (RNNs) are a denomination of artificial neural networks where connections among nodes lay out a directed graph along the temporal sequence. Unlike feedforward neural networks, RNNs have the ability to use their internal state for processing the sequences of inputs. RNN is designed to recognize sequences, for example, a speech signal or a text [9]. (iii) Recursive neural networks are more like a hierarchical network where there is really no time aspect to the input sequence, but the input has to be processed hierarchically in a tree fashion [8, 10]. Generally, different external stimuli match to different brain activities, and the different brain activities display different functional brain images [11]. For that, image classification plays a significant role in identifying different activities of the brain. Recently, many methods of deep learning were proposed to perform classification of image for different brain activities [12, 13]. To identify different activities of the brain including emotions, motor, social, relational and language activities, and working memory, Koyamada et al. [12] applied a feedforward deep neural network from images of functional magnetic resonance imaging (fMRI) to implement this mission. The feedforward deep neural network involved a softmax layer and multiple hidden layers. Similarly, these hidden layers were used to get high-level latent features, while the softmax layer was applied to calculate the probability of every subjects in a class. In addition, dropout, minibatch stochastic gradient descent, [14], and principal sensitivity analysis [15] were combined into the feedforward deep neural network to improve the performance of the final classification. Recently, to classify different sensorimotor tasks including auditory attention, visual stimulus, right-hand clenching, and left-hand clenching, Jang et al. [13] used fully connected feedforward deep neural networks and multiple hidden layers. In addition to the above classifications, the methods of deep learning classification of magnetic resonance imaging (MRI) images have been used also by other fields of classification, like stroke diagnosis [16], age prediction [17], classification of attention deficit hyperactivity disorder (ADHD) [18], discrimination of cerebellar ataxia types [19], and emotional response prediction [20]. Due to the science engineering field, it was doable to create systems of computer-aided diagnosis (CAD) that play a critical role in assisting the researchers and physicians when they interpret the medical imaging. Recently, the use of the machine learning approach, especially DL techniques in systems of CAD to diagnose and classify the healthy control normal (CN) people, Alzheimer's disease (AD), and mild cognitive impairment (MCI) patients, has exponentially increased [21, 22]. The Alzheimer's disease automatic diagnosis, especially in its early stage, plays a significant role in human health. Since Alzheimer's disease is a neurodegenerative illness, it has a long period of incubation. Thus, it is necessary to analyze the AD symptoms at different stages. Currently, a lot of researchers have proposed using the classification of images to perform diagnosis of AD. Moreover, many DL methods have been proposed to implement severity classification of different Alzheimer's disease patients by using MRI images [22, 23]. As known in image processing and analyzing, the better the image quality, then the better the results gained. However, the image quality depends on acquisition of the image, so, when the image acquisition is better, then the image quality is higher. Magnetic resonance imaging (MRI) not only keeps the features of noninvasive and good soft tissue contrast, but in addition does not expose humans to high ionizing radiation. Since MRI can provide a lot of invaluable information about structures of tissue, such as localization, size, and shape, it is attracting more of attention for computer-aided diagnosis and clinical routine [24, 25]. MRI can be divided into functional and structural imaging. Functional imaging contains tasking state functional MRI (ts-fMRI), resting state functional MRI (rs-fMRI), etc., structural imaging contains T1-weighted MRI (T1w), diffusion tensor imaging (DTI), and T2-weighted MRI (T2w) [26]. Medical data systems are diagnostic, and analytical systems are applied to help medical centers and physicians in disease treatment, and they are critical to improve treatment and diagnosis. Computer scientists have been interested in this domain given the vital role of medical data in the lives of humans. Physicians may refer to the classification of medical data, including medical analyses and symptoms of critical diseases, for making the decisions. A data set of disease contains symptoms of patients as attributes besides the number of instances of these symptoms. Health care may use the considerable medical data accessible. In the analyses of medical centers, data mining could be used to provide sufficient sources on illnesses for their prevention and timely detection and to avoid the expensive costs incurred by medical tests [27]. Representation of features plays a significant role in medical image analysis and processing. Deep learning has two obvious advantages in the representation of features:

- It can be applied to automatically discover features from a given data set for every specific application. Usually, methods of traditional feature extraction are based on some prior knowledge for extracting features in a certain application. So, these approaches are semiautomatic learning methods
- It can discover new features that are appropriate to specific applications, which have never been discovered by researchers previously. Traditional methods of feature extraction are often restricted by some a priori knowledge, which can only extract some features which are associated with a certain application [28, 29]

Medical imaging is the mechanism and process of establishing visual representations of the interior of the body for medical intervention and clinical analysis [30]. Machine learning tools and medical image processing can help neurologists in estimating whether a subject is developing Alzheimer's disease [31]. Alzheimer's disease is a chronic neurodegenerative disease causing tissue loss throughout the brain, and the death of nerve cells usually starts slowly and worsens over time [32]. Alzheimer's disease is expected to affect more and more people by the year 2050. The cost of caring for patients of AD is also expected to rise [33]. Presently, AD is the sixth reason that leads to death in the United States [34]. For this reason, individual computer-aided systems are necessary for accurate and early diagnosis of this disease [33]. There are many approaches for accurate and automatic classification of brain MRI, and one of them is our work. The next part of this article is the related works, then we will talk about our methodology, the results, the discussion, and, at the end, our references.

## 2. Related Works

Researchers have been applying machine learning techniques to build classifiers by using clinical measures and imaging data for AD diagnosis. These studies have identified the important structural differences in the regions such as the entorhinal cortex and hippocampus entorhinal cortex between the brain with AD and healthy brain. Different imaging methods like the functional and structural magnetic resonance imaging (fMRI and sMRI, respectively), single photon emission computed tomography (SPECT), position emission tomography (PET), and diffusion tensor imaging (DTI) scans which can perceive the changes causing AD due to the degeneration of cells of the brain. In recent years, deep learning models, especially convolutional neural networks, have demonstrated outstanding performance for medical image analysis. Payan and Giovanni [35] produced and tested a pattern classification system which combines convolutional neural network and sparse autoencoders. Ehsan et al. [36] adapted a 3D-CNN model for diagnosis of AD. The 3D-CNN is built upon the 3D convolutional autoencoder, which is pretrained to catch anatomical shape variations in scans of structural brain MRI. Sergey et al. [37] proposed two different kinds of 3D convolutional network architectures to classify the brain MRI which are the amendments of residual and plain convolutional neural networks. Applied convolutional neural networks can tackle the two problems stated before. These networks can propagate local features into the metarepresentation of an object for classification or image recognition. In deep learning for image classification, modern advancements like residual network architectures and batch normalization mechanism alleviate the issues of having small data sets of training, while providing a frame for automatic feature generation. As a result, these models can be used to 3D MRI images in the absence of intermediate handcrafted feature extraction. Karim et al. [38] adapted three tasks of binary classification which are considered for separating the normal control (NC) subject from mild cognitive impairment (MCI) patients and Alzheimer's disease (AD). Two fusion methods on a fully connected (FC) layer and on the single-projection CNN output offer better achievement by about 91% accuracy. The outcomes are competitive with the SOA which utilizes a heavier algorithmic chain. Fan and Manhua [39] proposed a classification technique built on multiple clusters of dense convolutional neural networks (DenseNets) to pick up the various local features for images of the MR brain, which are collected for classification of AD. The total brain image is partitioned into different local parts and from each region, a number of 3D patches are extracted. By using the*K*-means clustering method for grouping the patches from each region into different clusters, the DenseNet had been constructed to pick up the patch features for each cluster, and the features learned from the characteristic clusters of each part are grouped for classification. The classification outputs from different local parts are combined to foster the final image classification. This method can progressively learn the features of MRI from the local patches to the global image level for the task of classification. For preprocessing images of MRI, there are no segmentation and rigid registration required. Shaik and Ram [40] provided an approach to extract the gray matter from the human brain and make the classification by using the CNN. To enhance the voxels, a Gaussian filter is applied, and to remove the irrelevant tissues, the skull stripping algorithm is used. After that, by applying a hybrid, enhanced, and independent component analysis, those voxels are segmented. The input to the CNN was segmented gray matter. Clinical valuation was performed using the provided approach and 90.47 accuracy was achieved. Hamed and Kaabouch [41] proposed a method that yielded good classification accuracy. The convolutional neural network with modified architecture was used to get the high quality features from the brain MRI to classify people into healthy, early mild cognitive impairment (EMCI), or late mild cognitive impairment (LMCI) groups. The results showed the classification between control normal (CN) and LMCI groups in the sagittal view with 94.54 accuracy.

## 3. Materials and Methods

Inside a CNN, a filter series, with an equivalent size to a small image patch, automatically searches the entire image to find images of similar spatial features. These filters can be learned and updated independently; thus, a collection of them can detect crucial information of a specific task and data set [42]. There are standard steps of CNN. The first step is named “convolution”; this step is responsible for finding the features and applying filters. It is a filter kernel that picks up its weights by convolving the input data tensor with such kernel. There are several variables that effect the convolutional operation output such as strides and number of filters. The distance in pixels between two pixels is the stride, while the number of filters states the output feature map number [43]. The operation of convolution is just a mathematical operation, which should be treated equally with other operations such as multiplication or addition and should not be discussed particularly in the literature of machine learning. But, it has still been discussed here for completeness. Convolution is a mathematical operation on two functions (e.g., *f* and *g*) and produces a third function *h*; this is an integral that expresses the amount of overlap of one function (*f*) as it is shifted over the other function (*g*) [44]. Formally, it is described as

(1) $$\begin{array}{c} h\left(t\right)=\int_{-\infty }^{\infty }f\left(T\right)g\left(t-T\right)dT, \end{array}$$

And denoted as *h* = *f*∗*g*.

A typically convolutional neural network works with two-dimensional convolution operation that could be summarized in Figure 1. As displayed in Figure 1, the input matrix is Figure 1(a), and Figure 1(b) is usually called a kernel matrix. So convolution is applied to these matrices, then the result is displayed as in Figure 1(c). The process of convolution can be considered as an element-wise product followed by a sum, like what is shown in the example of Figure 1. When the left upper matrix which is 3 × 3 convoluted with the kernel, then the result is 29. After that, the target 3 × 3 matrix slides one column to the right, then is convoluted with the kernel and gets the result 22. The sliding and recording of the results have been continued as a matrix. Every target matrix is 3 × 3, because the kernel is 3 × 3; thus, the whole 5 × 5 matrix is shrunk into a 3 × 3 matrix when every 3 × 3 matrix is convoluted to one digit. (Because of 5 − (3 − 1) = 3, the first 3 means the kernel matrix size.) One should realize that the convolution process is a locally shifted invariant, which means that for many different combinations of how the nine numbers in the upper matrix 3 × 3 are placed, the convoluted result will be 29. This invariant property plays a crucial role in vision problem because the result of recognition should not be changed due to shift or rotation of features in an ideal case. This crucial property is applied to be solved elegantly by [45], but CNN brought the performance up to a new level.

With each convolution layer, there is an activation function; the activation is an operation which converts the input from a linear data tensor to a nonlinear data tensor. In deep learning, many activation functions are popular such as rectified linear units (ReLU), sigmoid, and tanh [46]. Recently, the rectified linear unit (ReLU) has been used more than the other nonlinear functions, because it does not activate all the neurons at the same time [24]. The second step is named “Max Pooling”; this step is responsible for downsizing the image and keeping the important features. Pooling is the operation of downsampling which can be performed globally or locally. The function of global pooling returns for every 2D feature map a scalar value. The function of local pooling downsamples local image parts by a factor [43]. The third step named “flattening” converts to one dimension array (vector). The fourth step is named “full connection”; this step is responsible of building all needed connections. The fully connected layer (FC) is typically followed by an activation layer. FC is the layer where the receptive domain is a whole channel of the former layer [43, 46]. The last step is named “classifier”; it represents the classification stage to decide if the image is normal or abnormal [47]. The use of the dropout technique is so common in convolutional neural networks. Dropout was introduced in [14, 48]. This mechanism soon got influential, not only because it has good performance but also because of its simplicity of implementation. The idea is very easy: while training, randomly drop out some of the units. More formally: for each training case, every hidden unit is randomly omitted with a probability of *p* from the network. As suggested in [14], dropout can be seen as an efficient method to perform model averaging across a great number of different neural networks, where overfitting can be avoided with less cost of computation because of the actual performance which it introduces. Dropout became very popular upon when it was first introduced; many works have attempted to understand its technique in different perspectives, including [49]. It has also been used to train other models, such as SVM [50].

The CNN architecture which was used in this study is composed of five convolutional layers which take an input image (the brain's MRI slice) with a size of 200∗200.  Figure 2 shows some slices of the brain's MRI; those were we used in our research. All five convolutional layers were followed by a max-pooling layer. The 64 filters with a kernel size of 9∗9 were considered for the first convolutional layer, and the max-pooling layer kernel size was set on 2∗2. The 64 filters with a kernel size of 7∗7 were considered for the second convolutional layer, and the max-pooling layer kernel size also was set on 2∗2. The 64 filters with a kernel size of 5∗5 were considered for the third convolutional layer, and the max-pooling layer kernel size was set on 2∗2. The 32 filters with a kernel size of 5∗5 were considered for the fourth convolutional layer, and the max-pooling layer kernel size was set on 2∗2.The 32 filters with a kernel size of 3∗3 were considered for the fifth convolutional layer, and the max-pooling layer kernel size was set on 2∗2. It is worthwhile to mention that the ReLU (rectified linear unit) function was used as the activation functions in all convolutional layers. The ReLU function is used commonly in models of DL; basically, if the function receives a negative value as input, it returns 0, and if the function receives a positive value, then the same positive value will return.

The function of ReLU is understood as *f*(*a*) = max(0, *a*).

Figure 3 demonstrates the block diagram of the proposed system (AlzNet). After the convolution layers and the flattening layer, there is a dense unit 121, and here, we used a ReLU as an activation function, then we used a dropout (0.2) to prevent overfitting, then there is a dense unit and sigmoid as an activation function; at the last stage, there is a binary classifier for displaying the results.

Table 1 demonstrates the number of MRI slices. There are samples for men and women such as a left-handed man (L.-handed male), left-handed woman (L.-handed female), right-handed man (R.-handed male), and a right-handed woman (R.-handed female); all brain MRIs were in the axial view manner. Keras provides a perfect tool to show a model's summary; Table 2 demonstrates that summary. This displays the number of trainable parameters and the output shape for each layer. Before starting to fit the model, this is a sanity check. So the total params = 414,419, the trainable params = 414,419, and the nontrainable params = 0.

## 4. Results

Python language 3.6 and Keras have been used for programming this work. Keras is a high-level library; it is an open source machine learning library that is written in Python. Keras is used for numerical computation purposes; it is used to perform the computations more easily and efficiently in practice. The training data set was 75% and the validation data set was 25%. There were many practical experiments that had been done in this research for trying to find the best parameters of this convolutional neural network. So we try to find the best number of dense units for hidden layers depending on the result of accuracy, whereas the other researches used different numbers at each one. Another parameter we tested many times is the rate of dropout to find the fit rate for our convolutional neural network by observing the results of accuracy. That is figured out in Table 3.

So it is obvious from Table 3 that the highest accuracy value was when we utilized 0.2 for the dropout rate and 121 for the dense unit. In fact, the range of the dropout rate which we tested was (from 0.1 to 0.5) increasing by 0.1, when the number of dense units was 120, 121, 122, 123, 124, 125, 126, 127, 128, 129, and 130.  Figure 4 shows the accuracy value depending on the relationship between the dense unit number and the dropout rate.

There are several metrics for measuring the performance of binary classification [51], such as recall, precision, specificity, and Accuracy. Precision is very helpful because we want to be confident of our forecast, since it tells us how many of the values expected as positive are actually positive [50], as follows:

(2) $$\begin{array}{c} \text{Precision}=\frac{\text{True positive}}{\text{True positive}+\text{False positive}}. \end{array}$$

Recall (sensitivity) is another very valuable measure that helps one, for instance, to know the proportion of the number of values accurately labeled as positive on the overall values which are actually positive, as follows:

(3) $$\begin{array}{c} \text{Recall}=\frac{\text{True positive}}{\text{True positive}+\text{False negative}}. \end{array}$$

Using the F1 score is a safe way to get a complete impression of recall and precision. The F1 score provides us the harmonic mean of recall and precision [52, 53], as follows:

(4) $$\begin{array}{c} \text{F}1\text{ score}=2*\frac{\text{Precision}*\text{Recall}}{\text{Precision}+\text{Recall}}. \end{array}$$

Accuracy is the proportion of accurate predictions (both true negative and true positive) among the entire number of cases examined [52], as follows:

(5) $$\begin{array}{c} \text{Accuracy}=\frac{\text{ True Positive}+\text{True Negative}}{\text{True positive}+\text{True negative}+\text{False positive}+\text{False negative}}. \end{array}$$

In this work, the measure metrics have been applied on the training data set and test data set (see Table 4).

## 5. Discussion

For our current work, we develop an efficient deep convolutional neural network based on a classifier and demonstrate very good performance by using the OASIS data set [54]. The OASIS-3 data set has been saved in the XNAT central repository [55]. In our work, a total of 15,200 MRI axial slices were used. The data was used to include the MRI scans of about 170 AD patients and 70 NC. They are all from different subjects that make the test of recognition performance more reliable. The age of each patient is between the range of 65-90 years old, both male and female in this work. At the first stage of data preprocessing, we obtained 2D slices from each MRI image. Then, the every last 20 dark slices with each time course was discarded because they included no functional information. Preprocessed images are augmented by rotating the slices to see whether or not the model can recognize the images; this increased the samples size and made a good training of the CNN model. The scans are T1-weighted whereas those of [40] were T2-weighted. Whereas [35, 41] used three convolution layers, our proposed system (CNN model) has 5 convolution layers; each convolution layer has ReLU as an activation function. Each convolution layer is followed by max pooling layers. Our proposed approach performs binary classification to fit the model in a batch size of 64 in 150 epochs.  Table 2 summarizes the total architecture of the proposed system. When [40, 41] used Adam optimization, we trained the model by Adadelta optimization with a dropout rate of 0.2 for the dropout layer which had been utilized to prevent the overfitting like in [40], but [41] used a 0.5 dropout rate. The number of dense units was 121 when the number of dense units of [37] was 128; actually, we made many experiments to decide which is the best number of dense units we should take, and Table 3 shows that. In this work, we tried to put different values of the neural network parameters by trial and error, by relying on the accuracy value, and comparison with previous researches. During binary classification, we trained the classifier for AD and CN images, and the model resulted in 97.88% training accuracy and 99.30 test accuracy. It is required to mention that our proposed framework had been trained, and the prediction was made with utmost accuracy.  Figure 5 demonstrates that. The accuracy of the proposed system has been compared with different models discussed in literature reviews as shown in Table 5.

It is observed that the proposed model achieves remarkable performance. The last thing we have to say is that neural networks have plenty of parameters, and any change in one of them will make the value of results different, and also, there is a big important reason for making a variation of results—it is the data set and its type.

## 6. Conclusions

In order to diagnose Alzheimer's disease, deep neural networks, especially CNNs, can provide meaningful information. A CNN-based method for extracting discriminatory features from structural MRI was proposed in this paper, with the goal of classifying Alzheimer's disease and healthy subjects using 2D MRI slices. For potential AD individuals, the suggested approach can lead to many advantages and can also lead to an early diagnosis of AD. The experimental results of the OASIS database for 240 subjects demonstrated that our proposed method of extraction and classification of features provided high accuracy for AD and CN. The best results have been obtained for the classification between the CN and the AD axial view of the MRI. The proposed method yielded a classification accuracy of 99.30 percent. The above results indicate higher reliability, recall, precision, and F1 score of our proposed method for the diagnosis of AD and the classification between CN and AD.

## Figures and Tables

**Figure 1:** A simple illustration of a two-dimension convolution operation: (a) input matrix, (b) kernel matrix, and (c) output matrix after convolution.

**Figure 2:** Some brain MRI slices of Alzheimer's patients.

**Figure 3:** Block diagram of proposed system (AlzNet). There are five convolutional layers; after each convolutional layer there is a max-pooling layer; the activation function in every convolutional layer was ReLU. After the convolution layers and flattening layer, there is a dense unit 121 with a ReLU as an activation function, with a dropout to prevent overfitting, then there is a dense unit and sigmoid as an activation function; at the last stage, there is a binary classifier.

**Figure 4:** Accuracy of AlzNet depending on dropout rate and dense unit.

**Figure 5:** Measure metrics of training data set and test data set.

**Table 1:** Number of MRI slices.

Subjects	Number of subjects	Number of MRI slices
R.-handed male (AD patient)	60	3050
L.-handed male (AD patient)	40	2600
L.-handed female (AD patient)	30	2150
R.-handed female (AD patient)	40	2600
Female (NC)	25	2000
Male (NC)	45	2800

**Table 2:** Summary of the proposed model.

Layer (type)	Output shape	Param #
Conv2d_1 (Conv2D)	(None, 192, 192, 64)	15,616
Max_pooling2d_1 (MaxPooling2)	(None, 96, 96, 64)	0
Conv2d_2 (Conv2D)	(None, 90, 90, 64)	200,768
Max_pooling2d_2 (MaxPooling2)	(None, 45, 45, 64)	0
Conv2d_3 (Conv2D)	(None, 41, 41, 64)	102,464
Max_pooling2d_3 (MaxPooling2)	(None, 20, 20, 64)	0
Conv2d_4 (Conv2D)	(None, 16, 16, 32)	51,232
Max_pooling2d_4 (MaxPooling2)	(None, 8, 8, 32)	0
Conv2d_5 (Conv2D)	(None, 6, 6, 32)	9248
Max_pooling2d_5 (MaxPooling2)	(None, 3, 3, 32)	0
Flatten_1 (flatten)	(None, 288)	0
Dense_1 (dense)	(None, 121)	34,969
Dropout_1 (dropout)	(None, 121)	0
Dense_2 (dense)	(None, 1)	122

**Table 3:** Accuracy of AlzNet depending on dropout rate and dense unit.

	Dropout rate					
		0.5	0.4	0.3	0.2	0.1
Dense unit	130	94.90	94.21	94.78	94.02	94.12
	129	95.18	95.72	95.61	95.31	95.48
	128	94.85	94.56	94.71	94.65	94.58
	127	95.09	95.12	95.01	95.23	95.31
	126	96.61	96.72	96.40	95.97	96.01
	125	96.15	96.05	96.11	96.44	96.21
	124	96.09	96.12	96.02	96.30	96.05
	123	95.91	95.72	95.82	95.01	95.11
	122	96.85	96.56	96.90	95.77	95.83
	121	97.32	97.16	97.30	97.88	97.06
	120	95.43	95.66	94.94	94.88	94.90

**Table 4:** Measure metrics of training data set and test data set.

Dataset	Precision	Recall	F1 score	Accuracy
Training	97.06	97.99	97.52	97.88
Test	98.92	99.53	99.22	99.30

**Table 5:** Literature reviews.

Methods	Year	Accuracy
Sergey et al. [37]	2017	80.00
Fan and Manhua [39]	2018	89.5
Shaik and Ram [40]	2019	90.47
Ehsan et al. [36]	2016	97.6
Karim et al. [38]	2017	91.41
Payan and Giovanni [35]	2015	95.39
Hamed and Kaabouch [41]	2019	94.54
Proposed method	2020	99.30

## Data Availability

Our data set was from the OASIS database; the website is https://www.oasis-brains.org. The OASIS-3 data set has been saved in the XNAT central repository; the website is https://central.xnat.org.
